# Down-regulation of LINC00472 promotes osteosarcoma tumorigenesis by reducing FOXO1 expressions via miR-300

**DOI:** 10.1186/s12935-020-01170-6

**Published:** 2020-03-30

**Authors:** Jingwei Zhang, Jieyuan Zhang, Dong Zhang, Weifeng Ni, Haijun Xiao, Bizeng Zhao

**Affiliations:** 1 Department of Orthopedics, Shanghai Fengxian District Central Hospital/Southern Medical University Affiliated Fengxian Hospital, No. 6600 Nanfeng Road, Shanghai, 201499 China; 2 Department of Orthopedics, Shanghai Sixth People’s Hospital, No. 600 Yishan Road, Shanghai, 200233 China

**Keywords:** LINC00472, Osteosarcoma, FOXO1, miR-300

## Abstract

**Background:**

Osteosarcoma (OS) is one of the most common types of primary bone tumors which poses negative effects on the bones of both young children and adolescents. LncRNA LINC00472 has been reported to be involved with poor prognostics in breast cancer and ovarian cancer. As a new lncRNA, its role in OS remains to be elusive. Herein, we are focused to explore its regulatory mechanism in the development of OS.

**Methods:**

qRT-PCR was utilized to examine the expressions of LINC00472 and miR-300 in OS tissues and cell lines. OS cell lines of U2OS and MG63 were used to investigate the biological function of LINC00472. Xenograft tumor model was built in nude mice with MG63 cells.

**Results:**

The expressions of LINC00472 were inhibited in OS tissues and cells, and were negatively related to the expressions of miR-300. LINC00472 directly targeted miR-300. FOXO1 was inhibited in OS tissues and its expressions were negatively related to the expressions of miR-300. LINC00472 over-expressions decreased cell proliferation abilities and colony formation abilities. These effects were mediated by miR-300. The silence of LINC00472 and over-expressions of miR-300 suppressed FOXO1 expressions. LINC00472 greatly reduced tumor growth in vivo and this effect was attenuated by miR-300 mimic.

**Conclusions:**

From all the experiments and observations, we demonstrated that LINC00472 could be a potential tumor suppressor in OS through interacting with miR-300 and FOXO1.

## Background

Osteosarcoma (OS) is one of the most common types of primary bone tumors which poses negative effects on the bones of both young children and adolescents [1, 2]. Scientists have developed many treatment methods, including tumor sections, chemotherapies, and radiotherapies [3, 4]. However, the prognosis of OS patients is rather poor, and the 5-year survival rate of OS patients is still not satisfied. The underlying reason might be the complex and complicated molecular mechanism of OS tumorigenesis [5, 6]. Therefore, it is necessary to discover new targets for the diagnosis, treatments, and prognosis of OA to improve patients’ survival and life quality.

Long non-coding RNAs (lncRNAs, > 200 nt) are groups of RNAs that do not code for proteins [7, 8]. In recent years, lncRNAs have been attracting more and more interest in the tumorigenesis and progression in many kinds of human cancers such as pancreatic cancer [9], gastric cancer [10], cervical cancer [11]. For OS, there are also many lncRNAs that were proved to play essential roles in the tumor development for OA patients. For instance, CL. Zhang reported that antisense lncRNA FOXC2-AS1 promoted doxorubicin resistance in OS by increasing the expressions of FOXC2 [12]. Wang revealed that LINC00161 sensitized OS cells to cisplatin-induced apoptosis by regulating the miR-645-IFIT2 axis [13]. LncRNA LINC00472 has been reported to be involved with poor prognostics in breast cancer [14] and ovarian cancer [15]. As a new lncRNA, its role in OS remains to be elusive. Herein, we are focused to explore its regulatory mechanism in the OS.

MicroRNAs (miRNAs) are another group of non-coding RNAs with a length of 20–23 nt [16, 17]. Previous researchers have demonstrated a series of miRNAs that participate in the regulation of OS. For example, Xue revealed that the up-regulation of miR-300 promoted proliferation and invasion of OS by targeting BRD7 [18]. In our preliminary experiments on bioinformatics, we found that LINC00472 could target miR-300. The expressions of forkhead box (FOX) proteins in OS are critical and closely involved in the development and progression of OS [19]. Our preliminary bioinformatics also indicated that miR-300 may interact with FOX-1 in OS. Therefore, we will study the associations among LINC00472, miR-300, and FOX-1 in OS development.

## Methods

### Clinical samples

From 2010 to 2012, we got OS tissues and matched normal tissues from patients who underwent surgeries in our hospital. OS patients included 13 males, 7 females, with an average age of 14.6 ± 4.18 years’ old, and ranged from 8 to 26 years’ old. The research was approved by the Ethics Board at Southern Medical University Affiliated Fengxian Hospital. The study followed the protocol of the Declaration of Helsinki. We explained the nature and possible consequences of the study to the participants, and informed written consent was obtained from them.

### Cell culture

The human normal osteoblast cell line of HFOB1.19 and OS cell lines of KHOS, MG63, U2OS, HOS, and Saos-2 were provided by Bank of Type Culture Collection of Chinese Academy of Sciences, China. HFOB1.19 cells were maintained in F12 with 10% FBS. HOS cells were cultured in Eagle’s minimum essential medium. Other cells were maintained in RPMI-1640 with 10% FBS. The medium and FBS were provided by Gibco, USA. Cell incubation was performed at 37 °C with 5% CO_2_.

### Cell transfection

A LINC00472 transcript (2933 bp, NR_026807.1) was assembled and inserted in a lentiviral vector, pCDH-EF1-MCS-pA-PGK-copGFP-T2A-Puro (pCDH), as previously described [14]. The sequence of the insert has been confirmed by sequencing. LINC00472 or FOXO1 were inserted to pCDH or pcDNA3.1 (GenePharma, China) for LIC00472 over-expression or FOXO1 over-expression, respectively. shNC, pCDH-vector, miR-300 mimic, and miR-NC (GenePharma, China) were also transfected into the cells via Lipofectamine 3000.

### qRT-PCR

RNAs were extracted via TRIzol reagent (Invitrogen, Carlsbad, CA). Subsequently, the reverse transcription reaction was performed for total RNA via cDNA Synthesis Kit (Thermo Fisher Scientific, USA). SYBR Green I Kit (Roche, UK) was utilized for RT-qPCR. The samples were subjected to qPCR in a real-time fluorescence qPCR (ABI7500, Applied Biosystems, Foster City, CA, USA). The results were calculated via 2^−ΔΔ*C*t^. The primer sequences were: LINC00472 forward GATGGCAGCTGTCTCTCTCC; reverse: GGGCCTCTCTGACCGTATCT; FOXO1: Forward 5′-GGCTGAGGGlTrAGTGAGCA-3′; reverse 5′-AGGGAGTTGGTGA A AGACATC-3′; GAPDH: forward GTCAAGGCTGAGAACGGGAA; reverse: AAATGAGCCCCAGCCTTCTC; MiR-300: forward: 5′-TATACAAGGGCAGACTCTCTCT-3′; reverse 5′-GTGCAGGTTCCGAGGT-3′; U6: forward 5′-CTCGCTTCGGCAGCACATATACT-3′; reverse 5′-ACGCTTCACGAATTTGCGTGTC-3′.

### Luciferase reporter assays

The wild-type (WT) and mutant (MUT) reporter plasmids of LINC00472 (LINC00472-WT and LINC00472-MUT) and the WT and MUT reporter plasmids of FOXO1 (FOXO1-WT and FOXO1-MUT) were provided by Shanghai GenePharma (Shanghai, China). Cells had co-transfection with miR-300 mimics or miR-control and pMIR-reporter luciferase vector with LINC00472-WT or LINC00472-MUT and FOXO1 via Lipofectamine 3000. Cells were lysed for luciferase detection at 2 days after transfections. The luciferase activities were normalized to *Renilla* luciferase activities.

### Cell viabilities assay

For cell proliferation analysis, we seeded the cells onto 96-well plates at 3 × 10^3^ cells per well. After 2 h of incubation with the cell proliferation reagent (Roche Diagnostics GmbH), cell concentrations were measured at 0, 1, 2, 3 and 4 days of culture with optical density (OD) at 450 nm wavelength using a microplate spectrophotometer (Biotek Synergy 2).

### Migration and invasion assays

The 24-well transwell chamber, with or without Matrigel (Corning, USA) was used to detect cell migration and invasion rates, respectively. Cells were fixed with 100 ml of serum-free medium and seeded into the upper chamber. 500 ml of DMEM containing 10% serum was pipetted to the lower chamber. After 24 h of incubation, the cells attached to the lower surface of the upper chamber were treated with 4% paraformaldehyde, stained with crystal violet, and analyzed under a microscope. 5 fields of vision were randomly selected for each hole under the microscope for photographing, counting, and statistical analysis.

### Colony formation

Cells/well were incubated in DMEM containing 10% fetal bovine serum at 37 °C. After 14 days, cells were washed, fixed in methanol for 30 min, and stained with 1% crystal violet dye. Then, the cell colonies were measured.

### Western blotting

Proteins were isolated via NP40 lysate, electrophoresed in 10% SDS-polyacrylamide and transferred to polyvinylidene fluoride membrane (Millipore, USA). It was treated with anti-FOXO1 (1:500, ab52857, Abcam, UK) or anti-GAPDH (1:1000, Beyotime, China) at 4 °C for a night. The membranes were then incubated in secondary antibody for an hour at 25 °C. After washing, we detected the signal using the ECL kit (P0018, Beyotime, China).

### Xenograft mouse model

10^6^ MG63 cells were transfected with lv-sh-NC or lv-sh-SNHG1. Then, they were injected to 8-weeks’ old nude mice (n = 5 mice/group). The tumor volumes were detected every 7 days. All animal experiments were performed in the animal laboratory center of Southern Medical University Affiliated Fengxian Hospital, which is in accordance with the Guide for the Care and Use of Laboratory Animals (National Institutes of Health, Bethesda, MD, USA). The protocols were approved by the Animal Care and Use Committee of Southern Medical University Affiliated Fengxian Hospital.

### Immunostaining

After 28 days, mice were euthanized. Xenograft tumors were dissected out, fixed in 4% PFA, and embedded in paraffin. The paraffin areas were stained with anti-Ki67 antibody (Santa Cruz Biotechnology, USA).

### Statistical analysis

All data were shown as mean ± SD from 5 replicas. Statistical analysis was performed using SPSS 18.0 and GraphPad. Differences were considered significant if P < 0.05.

## Results

### LINC00472 was suppressed and miR-300 was up-regulated in OS tissues and cell lines

To examine the functions of LINC00472 in OS, LINC00472 expressions were detected in tumor and normal tissues from 20 patients with OS. The data demonstrated that LINC00472 expression was markedly lower in OS tissues than normal ones (P < 0.001) (Fig. 1a). miR-300 level was elevated in OS tissues than normal ones (P < 0.001) (Fig. 1b). Moreover, LINC00472 expressions had negative correlation with the expressions of miR-300 (Fig. 1c). In different OS cell lines, expressions of LINC00472 were suppressed and expressions of miR-300 were promoted, in contrast to normal tissues (Fig. 1d, e).

**Fig. 1:** LINC00472 was suppressed and miR-300 was up-regulated in OS tissues and cell lines. **a** Relative expressions of LINC00472 in OS tissues and adjacent normal tissues (n = 20). **b** A. Relative expressions of miR-300 in OS tissues and adjacent normal tissues (n = 20). **c** The relationship between LINC00472 and miR-300 expressions in OS tissues. **d** The expressions of LINC00472 mRNA levels in OS cell lines. **e** The expressions of miR-300 mRNA levels in OS cell lines. (*P < 0.001, n = 5)

### MiR-300 was regulated by LINC00472 in OS cells

It has been reported that lncRNA can modulate posttranscriptional regulation through interfering with miRNA. By searching StarBase v.2.0, we speculated that miR-300 may have putative binding sites with LINC00472 (Fig. 2a). To confirm that, a dual-luciferase reporter assays were carried out. The data revealed that expressions of miR-300 mRNA were promoted in MG63 and HEK293T cells transfected with miR-300 mimic (Fig. 2b). Luciferase activities of pMIR-REPOR-LINC00472-WT were reduced by miR-300 mimic, but the pMIR-REPOR-LINC00472-MUT activities were not changed in both MG63 cells and HEK293T cells (Fig. 2c). Furthermore, miR-300 level was found to be up-regulated after cells transfected with sh-LINC00472 (Fig. 2d). In contrast, over-expressions of LINC00472 decreased the expressions of miR-300 obviously (Fig. 2e).

**Fig. 2:** miR-300 was modulated by LINC00472 in OS cells. **a** The putative target sequence for miR-300 on the 3′-UTR of LINC00472. **b** The expressions of miR-300 mRNA levels in MG63 and HEK293T cells had transfection with miR-NC and miR-300 mimic. **c** The luciferase activities were detected by luciferase reporter assays. **d** The expressions of LINC00472 mRNA levels in MG63 and U2OS cells. **e** The expressions of miR-300 mRNA levels in MG63 and U2OS cells. *P < 0.05, n = 5

### The effects of LINC00472 were mediated by miR-300 in OS cells

To confirm whether LINC00472 affects OS cell lines, miR-300 mimic and pcLINC00472 were co-transfected into MG63 and U2OS cell lines. CCK-8 and colony formation assays showed that over-expression of LINC00472 was correlated with suppressed cell proliferation, whereas miR-300 mimic increased cell proliferation (Fig. 3a–c). A similar phenomenon was also observed in migration and invasion assays, in which miR-300 mimic greatly reversed pc-LINC00472 induced decrease in cell migration and invasive (Fig. 3d, e). Figure 3f demonstrated the Western blotting for the expression of PCNA, Ki67, and GAPDH in MG63 and U2OS cells transfected by control, pcLINC00472, or pcLINC00472 + mi-300 mimic. It is obvious that pcLINC00472 suppressed the expressions of PCNA and Ki67, but miR-300 mimic attenuated these effects in both MG63 and U2OS.

**Fig. 3:** The effects of LINC00472 were mediated by miR-300 in OS cells. **a** CCK8 assays. **b**, **c** Colony formation. **d**, **e** Transwell migration and invasion assays. F. Western blotting for the expression of PCNA, Ki67, and GAPDH in MG63 and U2OS cells transfected by control, pcLINC00472, or pcLINC00472 + mi-300 mimic. *P < 0.001, **P < 0.05, n = 5

### FOXO1 was a direct target of miR-300

Based on these results, we aimed at identifying the main target genes of miR-300, which was predicted by Starbase 2.0 and miRanda algorithms. FOXO1 was predicted to be a target of miR-300 (Fig. 4a). Thus, we performed reporter assays with a luciferase plasmid harboring the 3′UTR sequence of FOXO1 containing the predicted miR-300 binding site. Furthermore, we developed mutant reporter vectors FOXO1-MUT and wildtype reporter vectors FOXO1-WT. These plasmids had co-transfection into HEK293T cells and MG63 with miR-300 mimic. Reporter assays in 293T and MG63 cells revealed miR-300-dependent repression of the FOXO1-WT 3′UTR (Fig. 4b). Consistent with the reporter assays, FOXO1 protein expressions were decreased in the presence of miR-300 mimic in OS cells (Fig. 4c). In addition, FOXO1 levels increased after treatment with pc-LINC00472 and decreased after treatment with sh-LINC00472 (Fig. 4d). These results indicate that FOXO1 was a direct target of miR-300.

**Fig. 4:** FOXO1 was a direct miR-300 target. **a** The putative target sequence for miR-300 in the 3′-UTR of FOXO1. **b** The luciferase activities were detected by luciferase reporter assays. **c** The expressions of FOXO1 protein levels in MG63 and U2OS cells had transfection with miR-NC and miR-300 mimic. **d** The expressions of FOXO1 protein levels in MG63 and U2OS cells. *P < 0.001, **P < 0.05 n = 5

### FOXO1 attenuated the effects of miR-300 mimic in OS cells

To determine whether FOXO1 was involved in the LINC00472/miR300 mediated OS cell proliferation and invasion, we performed rescue experiments. Figure 5a confirmed the successful transfection with FOXO1. OS cells had co-transfection with pcDNA-FOXO1 and miR-300 mimic. CCK8 (Fig. 5b), colony formation (Fig. 5c) and transwell assays (Fig. 5d) showed that pcDNA-FOXO1 partially reverse the miR-300-induced cell proliferation and migration. Figure 5e demonstrated the Western blotting for the expression of PCNA, Ki67, and GAPDH in MG63 and U2OS cells transfected by control, mi-300 mimic, or mi-300 mimic + pcDA-FOXO1. It is obvious that miR-300 mimic elevated the expressions of PCNA and Ki67, but pcDA-FOXO1 attenuated these effects in both MG63 and U2OS.

**Fig. 5:** FOXO1 attenuated the effects of miR-300 mimic in OS cells. **a** The expressions of FOXO1 mRNA levels in MG63 and U2OS cells had transfection with vector and pcDNA-FOXO1. **b** CCK8 assays. **c** Colony formation experiment results and the cell numbers. **d** Transwell migration and invasion assays, and the cell numbers. **e** Western blotting for the expression of PCNA, Ki67, and GAPDH in MG63 and U2OS cells transfected by control, mi-300 mimic, or mi-300 mimic mi-300 mimic + pcDA-foxo1. *P < 0.001, **P < 0.05, n = 5

### Over-expressions of LINC00472 restrained growth of tumors by sponging miR-300 in vivo

To investigate if LINC00472 regulated OS by interacting with miR-300, MG63 cell nude mouse xenograft model was established. The in vivo test was performed using a stable cell line. Mice were administered with MG63 cells in transfection with pc-LINC00472 and miR-300 mimic. Figure 6a–c displayed the tumor size was inhibited by LINC00474, but relieved by miR-300 mimic. Ki-67 was markedly suppressed by pc-LINC00472 from IHC analysis (Fig. 6d). Meanwhile, we found that the over-expressions of LINC00472 significantly promoted FOXO1 protein expressions level in vivo and this effect was attenuated by miR-300 mimic (Fig. 6e). A schematic diagram showing the relationship between LINCOO472, miR-300 and FOXO1 was presented in Fig. 7.

**Fig. 6:** Over-expressions of LINC00472 restrained tumor growth through targeting miR-300 in vivo. **a** Tumor volumes were detected every week, and growth curves were shown. **b** Tumor’s growth was inhibited in the sh-LINC00472 mouse compared with the control. **c** Tumor weight (g). **d** Ki-67 staining. **e** The expressions levels of FOXO1 in tumor tissues. *P < 0.001, **P < 0.05, n = 5

**Fig. 7:** A schematic diagram showing the relationship between LINCOO472, miR-300 and FOXO1

## Discussions

Xue et al. reported that the expressions of miR-300 were up-regulated in OS [18]. In our experiments, we also noticed that miR-300 level was greatly elevated in cancer tissues than normal ones. However, we found that LINC00472 level was dramatically lower in cancer tissues than normal tissues. LINC00472 expressions were negatively correlated with miR-300. In cell lines, we observed a similar phenomenon. Similar to previous reports, it was well established that miR-300 was enhanced in OS tissues and cells. However, we found that LINC00472 expressions were inhibited in OS tissues and cells for the first time.

According to previous researchers, miR-300 could target with lncRNAs such as TUG1 in gallbladder carcinoma [20] and PTTG1 [21]. As far as we know, we are the first to investigate the interactions between miR-300 and LINC00472 in OS. From StarBase, it was revealed that miR-300 had putative binding sites with LINC00472. The dual-luciferase reporter assays also revealed that LINC00472-WT was reduced by the miR-300 mimic, but LINC00472-mut had no change. In addition, we found that miR-300 level was up-regulated in cells transfected with sh-LINC00472. Over-expressions of LINC00472 decreased miR-300 levels markedly, while miR-300 was regulated by LINC00472 in OS cells. All the evidence proved that miR-300 could bind with LINC00472 in OS, which is a new finding in the area of OS tumorigenesis.

FOXO1 was shown to be a targeted by several miRNAs in OS cells. For instance, H. Pei et al. found that miR-135b promoted proliferations and invasions of OS cells by sponging FOXO1 [22]. In 2015, H. Guan et al. found that FOXO1 could inhibit OS oncogenesis via Wnt/β-catenin pathway suppression [23]. In our experiments, the luciferase reporter assay in 293T and MG63 cells revealed miR-300-dependent repression of the FOXO1-WT 3′UTR. Moreover, FOXO1 protein expressions were decreased in the presence of miR-300 mimic in OS cells. As a supplement to OS tumorigenesis, we conclude that FOXO1 was a direct miR-300 target.

According to N. Jiang, lncRNA DANCR promoted tumor progressions and cancer stemness feature in OS by up-regulating AXL through inhibiting miR-33a-5p [24]. Inspired from previous findings, we also noticed that LINC00474, miR-300, and FOXO1 may function together in the regulatory of OS. From our results, the CCK8, colony formation, and Transwell assays showed that pcDNA-FOXO1 partially reverse the miR-300-induced cell proliferation and migration. FOXO1 attenuated the effects of miR-300 mimic in OS cells. In the in vivo experiments, over-expressions of LINC00472 greatly promoted FOXO1 protein expressions level and this effect was blunted by miR-300 mimic. As far as we know, we are the first to establish that over-expressions of LINC00472 restrained tumor growth through targeting miR-300 in vivo.

As a limitation, our study used inference from transiently transfected cells, which are conclusive only for 24-48 h. Beyond these time point, stable cell lines expressing gene can better increase the accuracy of the test. In our future work we plan to employ the stably transfected cells, and compare cell viability, colony formation and mouse xenograft with those from transiently transfected cells.

## Conclusions

From all the experiments and observations, we demonstrated that LINC00472 could be a potential tumor suppressor in OS through interacting with miR-300 and FOXO1.

## Data Availability

The datasets used and/or analyzed during the current study are available from the corresponding author on reasonable request.

## Abbreviations

OS: Osteosarcoma
miRNAs: MicroRNAs
lncRNAs: Long non-coding RNAs
FOX: Forkhead box
